This article has been retracted.

# Research on the Formation Mechanism of MgO and Al_2_O_3_ on Composite Calcium Ferrite Based on DA-RBF Neural Network

**DOI:** 10.1155/2022/4327969

**Published:** 2022-01-05

**Authors:** Baoliang Ma, Yuzhu Zhang, Lixing Ma

**Affiliations:** ^1^School of Metallurgy, Northeastern University, Shenyang 110819, China; ^2^School of Metallurgy and Energy, North China University of Science and Technology, Tangshan 063210, China; ^3^School of Qian'an College, North China University of Science and Technology, Tangshan 064400, China

## Abstract

Calcium complex ferrate is an ideal binder phase in the sintered ore phase, and a detailed study of the whole process of calcium complex ferrate generation is of great significance to improve the quality of sintered ore. In this paper, we first investigated calcium ferrate containing aluminum (CFA), which is an important precursor compound for the generation of complex calcium ferrate (SFCA), followed by a series of composite calcium ferrate generation process phase XRD detections and data preprocessing of data. Data correlation and data fitting analysis were combined with composite calcium ferrite phase diagram energy spectrum analysis to obtain the effect of MgO and Al_2_O_3_ on the formation of composite calcium ferrite. Then a modified RBF neural network model using the resource allocation network algorithm (RAN) was used to predict the generation trend of complex calcium ferrate. The parameters of the neural network are optimized with the Dragonfly algorithm, compared with the traditional RBF neural network. The prediction accuracy of the improved algorithm was found to be higher, with a prediction result of 97.6%. Finally, the predicted results were based on comparative metallurgical experimental results and data analysis. The validity and accuracy of the findings in this paper were verified.

## 1. Introduction

The ore-forming process of sinter is that some low-melting substances and low-melting substances produced by solid-phase reactions during the sintering process are melted into liquid phase under the action of high temperature, and the liquid phase solidifies in the subsequent cooling process to become the strong connection of solid particles that have not been melted and particles that have dissolved into the liquid phase [1]. Against the background of the utilization of low-quality raw materials faced by China's steel industry with large total output but increasingly depleted mineral resources, sinter mineralization research has important theoretical and application value in elucidating the sintering ore-forming mechanism and improving the metallurgical properties of sinter.

Many scholars have studied the metallurgical properties of sinter through metallurgical experiments and other metallurgical techniques. Zhang and others mixed ordinary magnetite concentrate and high-chromium vanadium-titanium magnetite raw materials and studied the influence of TiO_2_ mass fraction on the properties of high-chromium vanadium-titanium magnetite sinter through sintering experiments. The results show that, with the increase of TiO_2_ mass fraction, the transfer index gradually decreases in a certain range, and the strength of sintered ore decreases. The vertical sintering speed, yield, and sinter cup utilization coefficient show an increasing trend. The proportion of small particle size sintered ore with diameter less than 5 mm gradually decreases, and the particle size has a tendency to increase [2]; Du conducted a systematic quantitative study on the ore phase structure of sintered ores with different types of external ores as the main iron-bearing raw materials. The influence law of external ore on its mineral phase structure was analyzed. The quantitative relationship between the sinter phase characteristics and metallurgical properties was found, and the final results suggested that Newman's powder was the main raw material for iron content, accompanied by small amounts of Mike's powder, Yandy's powder, and superspecial powder to improve the quality of sintered ore [3]; Han et al. quantitatively studied the microstructures of two high-basic magnetite sinter through a polarized light microscope and, combined with metallurgical performance testing, discussed the influence of the sinter microstructure on its metallurgical properties. The results show that the large development of skeletal crystalline and granular hematite and the structural inhomogeneity make the second sintered ore significantly weaker than the first sintered ore in terms of resistance to low-temperature reduction pulverization, while the reduction of the second sintered ore is slightly better than that of the first sintered ore, which is related to the fact that the microstructure of the second sintered ore is dominated by large pores, and the pore rate is as high as 30% [4]; Yao used mineral phase microscope, XRD, SEM, and EDS to analyze the samples and studied the equilibrium phase composition of sinter with different aluminum content and the influence on the metallurgical properties of sinter. The results show that when the Al_2_O_3_ content in the sintered ore is increased, the aluminum solid solution complex calcium ferrate phase increases significantly, the magnetite phase and dicalcium silicate decrease, the aluminum content increases the fusibility temperature, the temperature interval becomes narrower, the strength becomes worse, and the reducibility improves [5].

In recent years, some scholars have also applied intelligent algorithms to basic research on the influence of sintering ore-forming behavior. Amin Anbaz et al. illustrated that the adsorption density on the structured activated carbon constructed by MLFNN in predicting CO_2_ is porous adsorption and ANN can estimate complex nonlinear functions; during the study the parameters of the proposed MLFNN (weight and bias) were optimized and these procedures were based on the differences between the outputs of the desired objectives [6]. Rostami et al. conducted a study including multilayer perceptual-artificial neural network (MLP-ANN) and radial basis function-artificial neural network (RBF-ANN) application including integrated modeling for accurate estimation of carbonate rock permeability in heterogeneous reservoirs; in addition the relevant parameters of MLP-ANN and RBF-ANN were optimized using ML and GA [7].Wang and Qiang combined the gray theory to weaken the volatility of data series and the advantages of neural network processing nonlinear adaptive information. Using the gray neural network model, only a small sample can be used to predict the alkalinity of sintered ore, but the prediction accuracy of the model is low and it is difficult to apply in practice [8]. Chen et al. established a prediction system for sintering chemical composition FeO and sintering yield based on BP neural network and obtained a high accuracy rate, but the model is old and lacks innovation [9]. Through the data visualization technology, Yang and Zhuansun studied the relationship between the various components of the pellet microstructure and the compressive strength and provided new research ideas for improving the compressive strength and metallurgical properties of the pellets [10] and achieved good results. Liu et al. designed a systematic RF framework based on random forest classification for lithium-ion battery manufacturing feature analysis and modeling, which simultaneously quantifies battery manufacturing feature importance and correlation through three different quantitative metrics, unbiased feature importance (FI), gain improvement FI, and PMOA, providing a model dimensionality reduction and effective sensitivity analysis for battery manufacturing [11]. Hu et al. used deep bidirectional long short-term memory (BiLSTM) to capture the periodicity (daily and seasonal patterns) of renewable energy generation and used residual techniques to improve the training efficiency of deep BiLSTM to develop a deep quantile prediction network (DQFN) based on IGD and deep residual BiLSTM for wind and solar quantile prediction [12]. Based on the above literatures, it can be seen that there are relatively few studies on the formation mechanism of MgO and Al_2_O_3_ in composite calcium ferrite using intelligent algorithms.

Composite calcium ferrite is an ideal binder phase in the sinter phase. Studying the formation reaction mechanism of composite calcium ferrite and increasing the content of composite calcium ferrite phase in the sinter phase have important theoretical guiding significance for enhancing the strength of the sinter, improving the reducibility, and improving the quality of the sinter. The research plans to use XRD to analyze the changes in the mineral phase content to infer the reaction sequence and analyze the substances in the sinter phase at each stage. The electron microscope was used to observe the magnesium-containing minerals and other mineral phases in the composite calcium ferrite phase area and to study the formation mechanism of composite calcium ferrite and the diffusion and migration behavior of MgO and Al_2_O_3_ during the sintering process.

Based on the above experiment of the influence of MgO and Al_2_O_3_ on the formation of composite calcium ferrite, the availability of data is analyzed, and the data set is optimized through data preprocessing methods. The data prediction model is used to predict the change trend of composite calcium ferrite formation under the influence of MgO and Al_2_O_3_. Furthermore, the results of composite calcium ferrite formation with the addition of different MgO and Al_2_O_3_ are summarized in an all-round and multilevel manner. The shortcomings of the existing prediction models are analyzed to improve the model and global optimization is performed on the center of gravity vector, width vector, and weight. Mutual verification with metallurgical experiment results in proving the applicability of neural network in the research of composite calcium ferrite.

## 2. Formation Mechanism of CFA in Al_2_O_3_-CaO-Fe_2_O_3_ System

Aluminum-containing calcium ferrite (CFA) is an important precursor compound for the formation of composite calcium ferrite (SFCA) [13]. It was found by extending the sintering time in the low-temperature solid-phase reaction stage: The starting temperature of C_2_F is less than 750°C; in the following reaction (1), the starting temperature of CF is between 750°C and 850°C, and reaction (2) is consistent with the research conclusion of Li et al. [14]. The formation temperature of CA2 is lower than the initial temperature of CFA (about 900°C); CA_2_ is formed at the C_2_F/Al_2_O_3_ interface, and the temperature is between 950°C and 1000°C. Therefore, the mechanism of CA_2_ formation is changed here. The formation reaction is as follows (3): CaO is generated by the decomposition of CaCO_3_; after that, CF, CA_2_, and Fe_2_O_3_ react to form CFA. Under the C_2_F-Al_2_O_3_-Fe_2_O_3_ ternary system, C_2_F-Al_2_O_3_ directly contacts and reacts to form CFA. However, in the solid state reaction of the CaO(CaCO_3_)-Al_2_O_3_-Fe_2_O_3_ ternary system, C_2_F is first formed at the CaO/Fe_2_O_3_ interface, the diffusion capacity of Fe^3+^ in CF is greater than that of Ca^2+^ in C_2_F layer, and CF is formed near the Fe_2_O_3_ particles at the C_2_F/Fe_2_O_3_ interface; the experimental results in the previous section show that the generation trend of CA_2_ is greater than that of CA. CA_2_ is formed at the CaO/Al_2_O_3_ interface. In the product layer around CaO, C_2_F and CA_2_ form the C_2_F/CA_2_ interface, but there is no C_2_F/Al_2_O_3_ interface or CF/CA_2_ interface. The schematic diagram of the reaction interface is shown in Figure 1. When the temperature is 850°C, C_2_F almost disappears, the C_2_F content decreases when the temperature rises, a large amount of CF is produced, and the C_2_F/CA_2_ interface transforms into the CF/CA_2_ interface. In addition, there is a large amount of Fe_2_O_3_ in the mineral phase, so the CFA formation reaction occurs, and CFA diffraction peaks appear at 850°C–900°C.

(1) $$\begin{array}{c} \text{CaO}+{\text{Fe}}_{2}{\text{O}}_{3}⟶{\text{C}}_{2}\text{F}\;\left(<750{}^{\circ}\text{C}\right), \end{array}$$

(2) $$\begin{array}{c} {2\text{Fe}}_{2}O_{3}+{\text{C}}_{2}\text{F}⟶\text{CF}\;\left(800{}^{\circ}\text{C}\right), \end{array}$$

(3) $$\begin{array}{c} {2\text{Al}}_{2}O_{3}+\text{CaO}⟶{\text{CA}}_{2}\;\left(900{}^{\circ}\text{C}\right), \end{array}$$

Analysis suggests that the CaO(CaCO_3_)-Al_2_O_3_-Fe_2_O_3_ ternary system first produces dicalcium ferrite C_2_F. Due to the interface limitation, C_2_F cannot directly react with Al_2_O_3_, and C_2_F transforms into ferrite monocalcium CF [15, 16]. At about 850°C, the CA_2_/CF interface appears, and CFA begins to slowly form. The reaction equation for its formation is CA_2_ + CF + Fe_2_O_3_ ⟶ CFA (850°C–900°C).

## 3. Phase XRD Detection of Composite Calcium Ferrite Formation Process

### 3.1. Phase Derivation of Al_2_O_3_-CaO-Fe_2_O_3_ Reactant

The XRD test results show that the integrated intensity changes of the diffraction peaks of each mineral phase are shown in Figure 2. At 750°C, a large amount of C_2_F exists and CF begins to form. The content of C_2_F decreases and disappears at 850°C; the content of CF first increases and then decreases and disappears at 950°C; around 900°C, the diffraction peaks of CA_2_ and CFA appear, which are lower than the formation temperature of the C_2_F-Al_2_O_3_-Fe_2_O_3_ ternary system; the integral intensity of CA_2_ and CFA gradually increased and began to decrease at 1050°C; the unknown substance X_2_ began to form at 1000°C and continued to increase. When the reaction of C_2_F-Al_2_O_3_-Fe_2_O_3_ and CaCO_3_-Al_2_O_3_-Fe_2_O_3_ ternary system is lower than 1000°C, the type of mineral phase and initial formation temperature are quite different. Compared with the test results of group B, the mineral phase of group A has CF. The temperature at which CA_2_ and CFA start to form decreases. After the temperature exceeds 1000°C, there is no significant difference in the change of the mineral phase content.

X-ray diffraction obtains the XRD pattern of the mineral phase. As the Al_2_O_3_ content increases from 1.5% (R7) to 3.5% (R11), the mineral phase is mainly composed of different forms of calcium ferrite, as well as a small amount of hematite and calcium aluminate, as shown in Figure 3.

Comparative analysis of the XRD diffraction peak intensity of different Al_2_O_3_ content found the following: (1) With the continuous increase of Al_2_O_3_ content, the intensity of the calcium ferrite C_4_F_7_ and Fe_2_O_3_ diffraction peaks in the mineral phase gradually weakened, and the diffraction peaks of other substances gradually increased [17]. Al_2_O_3_ solid-dissolves with calcium ferrite and can promote the dissolution of Fe_2_O_3_ in calcium ferrite to form composite calcium ferrite. Therefore, the content of Al_2_O_3_ increases, and the contents of Fe_2_O_3_ and calcium ferrite C_4_F_7_ gradually decrease, while the contents of composite calcium ferrite SFCA-I and CaAl_2_Fe_4_O_10_ gradually increase. (2) A large amount of Fe_2_O_3_ is solid-dissolved in the composite calcium ferrite, which leads to the molar ratio of CaO/Fe_2_O_3_>1 in the sintered ore, and the probability of contact between Al_2_O_3_ and CaO increases, which promotes the tendency of the diffraction peaks of C_2_F and CA_2_ to slightly increase. With the increase of Al_2_O_3_ content from 1.5% to 3.5%, the main mineral phase of the sintering phase changes from calcium ferrite to complex calcium ferrite.

### 3.2. XRD Detection under Different Temperatures and MgO Contents

With different MgO contents, different temperature sinter phase XRD detection results have different diffraction peaks [18, 19]; take w(MgO) = 1.3% as an example. The change trend of the integrated intensity of the mineral phase diffraction peaks of different MgO content experimental results is shown in Figure 4.

(1) For constant temperature sintering at 950°C for 2 hours, XRD did not detect dicalcium ferrite C_2_F and monocalcium ferrite CF diffraction peaks, as well as hemicalcium aluminate CA_2_, CFA diffraction peaks began to appear, and the integrated intensity gradually increased. It reaches the maximum around 1050°C–1100°C, and then the integrated intensity shows a downward trend and disappears at 1200°C. (2) Fe_2_O_3_ gradually decreases, showing a rapid downward trend around 1150°C. At the same temperature, the MgO content increases, while the Fe_2_O_3_ content shows a decreasing trend. (3) The integrated intensity of SiO_2_ diffraction peaks gradually decreases and disappears between 1175°C and 1200°C. As the content of MgO increases, the content of SiO_2_ increases with decreasing temperature, and the temperature decreases when it disappears. (4) With the increase of temperature, the integrated intensity of the diffraction peak of Ca_2_Mg (Si_2_O_7_) first increases and then decreases and increases with the increase of MgO content at the same temperature. When w(MgO) = 1.3%, the content of Ca_2_Mg(Si_2_O_7_) phase reaches the maximum value at 1000°C and then shows a downward trend, and the diffraction peak disappears at 1150°C. When w(MgO) = 2.6%, the content of Ca_2_Mg(Si_2_O_7_) phase reaches the maximum value at 1050°C and then shows a downward trend, and the diffraction peak disappears at 1175°C. When w(MgO) = 1.3%, the content of Ca_2_Mg(Si_2_O_7_) phase reaches the maximum at 1100°C and then shows a downward trend. The diffraction peak disappears at 1200°C. The MgO content increases, the Ca_2_Mg(Si_2_O_7_) content continues to increase, and the temperature range expands.

The formation content of magnesium-rich calcium ferrite (SFCAM) and the influence of its change trend are shown in Figure 5(d). The starting temperature of SFCAM is between 1000 and 1050°C, and the main generation temperature range is about 1150∼1225°C [20, 21]. As the temperature rises, the content of SFCAM composite calcium ferrite gradually increases; at 1250°C, SFCAM decomposes and the content decreases. As the temperature increases, the content of MgFe_2_O_4_ tends to increase. MgFe_2_O_4_ and Fe_3_O_4_ have similar crystal structures and have the same XRD diffraction peaks. MgO can promote the formation of Fe_3_O_4_ at 1100°C, and the high temperature decomposition of SFCAM to produce Fe_3_O_4_ increases the diffraction peaks. When the content of MgO increases and the temperature is lower than 1150°C, the content of complex calcium ferrite (initial generation content) shows a decreasing trend, which has an inhibitory effect on the formation of SFCAM. When the temperature exceeds 1150°C, the content of composite calcium ferrite increases, which promotes the production of SFCAM and can increase the production rate and content of SFCAM.

## 4. SFCAM Reaction Process Data Analysis

Affected by the sintering environment and human factors, there is a certain deviation between the SFCAM formation process phase XRD data detection, MgO and Al_2_O_3_ liquid phase formation kinetics experiment of the sintering system, and so forth and the true value. The stationarity test and preprocessing of the data can make the experimental results more convincing [22].

First of all, the data should be processed for outliers. Outliers refer to one or several values in the data which are quite different from other values [23]. The occurrence of outliers may be caused by the instability of the XRD data detection and other instruments and may also be caused by human operating errors. When there is a big difference between the detected data and other data, you can use the following: (1) Eliminate outliers and do not add observations; (2) eliminate outliers and add observations; or eliminate outliers and replace them with appropriate interpolation; (3) find out the actual reason and correct the outliers; otherwise, keep them [24]. These three methods carry out the preprocessing of abnormal data [25].

Before the outlier processing, it is necessary to detect the outliers [26]. The box plot method can be used to directly reflect the number and location of the outliers. Box plot drawing steps are as follows:

1. Draw the number axis, the unit is the same as the original unit, the starting point is slightly smaller than the minimum value, and the length is slightly longer than the full distance of the data batch.
2. Draw a rectangular box with the positions of the two sides corresponding to the upper and lower quartiles of the data batch; and draw a line segment at the median position inside the rectangular box as the median line.
3. Draw two line segments that are the same as the median line at *Q*_3_+1.5*σ*_*i*_ and *Q*_3_ − 1.5*σ*_*i*_. These two line segments are the outlier cutoff points, called the inner limit; draw two line segments at *Q*_3_+3*σ*_*i*_ and *Q*_3_ − 3*σ*_*i*_, and call them the outer limit. Outliers between the inner and outer limits are called mild outliers, and those outside the outer limits are extreme outliers.
4. Draw a line segment from both ends of the rectangular box to the farthest point that is not an outlier, indicating that the normal value distribution interval is within the data.

After preprocessing the data, through data correlation analysis (CCA) [27], the close degree of correlation between the components at different temperatures is obtained. Assuming that there are two sets of one-dimensional data sets *X* and *Y*, the correlation coefficient *ρ* is defined as follows [28]:

(4) $$\begin{array}{c} \rho \left(X,Y\right)=\frac{\mathrm{cov}\left(X,Y\right)}{\sqrt{D\left(X\right)}\sqrt{D\left(Y\right)}}, \end{array}$$

where cov(*X*, *Y*) is the covariance of *X* and *Y* and *D*(*X*) and *D*(*Y*) are the variances of *X* and *Y*, respectively.

Through Matlab simulation, the Kalman filtering method can control the influence of observations and abnormal state on parameter estimation and can effectively remove white noise [29].

Correlation analysis results show that the correlation coefficient between Fe_2_O_3_ and composite calcium ferrite SFCAM is −0.81, which has a great negative correlation. The correlation coefficient between Fe_2_O_3_ and Ca_2_Mg (Si_2_O_7_) is 0.75, which has a large positive correlation. The correlation analysis method is also applied to the influence of the MgO/Al_2_O_3_ ratio on the amount of liquid phase generated by sintering, which can further verify the correctness of the conclusion. The results show that the correlation coefficient between the ratio of MgO/Al_2_O_3_ and the amount of liquid phase produced by sintering is 0.86, which has a great positive correlation. In the previous studies on the influence mechanism of Al_2_O_3_ on the formation of calcium ferrite, the reaction mechanism of MgO on the formation of SFCAM, and the influence of Al_2_O_3_ on the amount and characteristics of sintering liquid phase formation, the data obtained are all discrete variables. In order to further describe and summarize the experimental results, a variety of fitting algorithms are compared on the basis of existing data [30], and the residual sum of squares is used as the evaluation standard. The comparison of fitting results is shown in Figure 6.

It can be seen from Figure 6 that the sum of squared residuals of the fourth-order polynomial is 0, which can better fit the hemispheric temperature change law with different Al_2_O_3_ content.

Combined with the analysis of the XRD detection mechanism of the calcium ferrite formation process, the analysis has reached the following conclusions: (1) The sintered sample was sintered at a constant temperature of 950°C for 2 hours through XRD detection. It was found that magnesium ferrite MgFe_2_O_4_ and calcium magnesium silicate Ca_2_Mg (Si_2_O_7_) (abbreviated as CMS) existed, indicating that reactions (5) and (6) had occurred. (2) The formation of CFA is detected in the temperature range of 950°C–1000°C. CFA is formed around the Al_2_O_3_ particles. The content of Al_2_O_3_ (5%) in the experimental raw material ratio is lower, so the generation temperature is higher than the experimental result in the previous section. (3) With the increase of CFA content, the MgFe_2_O_4_, Ca_2_Mg (Si_2_O_7_) phase content increases and slows down, and a small amount of composite ferrite SFCAM begins to form, indicating that CFA reacts with MgFe_2_O_4_, Fe_2_O_3_, and Ca_2_Mg (Si_2_O_7_) to form SFCAM; in formula (7), MgO mainly interacts with MgFe_2_O_4_ and Ca_2_Mg (Si_2_O_7_) to form magnesium-rich composite calcium ferrite. (4) When w(MgO) = 1.3%, when SFCAM starts to form and increases, there is a small amount of CFA in the mineral phase, and the amount of SFCAM produced at 1000°C–1100°C is less; the content of CFA in the mineral phase reaches the maximum at about 1100°C, and the content of SFCAM increases rapidly at 1100°C–1200°C. When the w(MgO) content is 1.6% and 3.9%, this phenomenon is also found, indicating that the increase of the CFA content in the mineral phase and the reaction of MgFe_2_O_4_, Ca_2_Mg(Si_2_O_7_), and Fe_2_O_3_ can promote the formation of SFCAM. Therefore, CFA is considered to be the key reactant for the formation of SFCAM from magnesium-containing minerals.

(5) $$\begin{array}{c} \text{MgO}+{\text{Fe}}_{2}{\text{O}}_{3}⟶{\text{MgFe}}_{2}{\text{O}}_{4}, \end{array}$$

(6) $$\begin{array}{c} {\text{SiO}}_{2}+\text{MgO}+\text{CaO}⟶\text{CMS}\;\left(\text{Calcium magnesium silicate}\right), \end{array}$$

(7) $$\begin{array}{c} \text{CFA}+\text{CMS}+{\text{MgFe}}_{2}{\text{O}}_{4}+{\text{Fe}}_{2}{\text{O}}_{3}⟶\text{SFCAM}, \end{array}$$

The content of w(MgO) increased from 1.3% to 3.9%. Both magnesium ferrite and magnesium calcium silicate can participate in the formation of composite calcium ferrite. The reaction mechanism of magnesium-containing mineral sintering during the formation of SFCAM is different. When the content of MgO is low, the content of MgFe_2_O_4_ and Ca_2_Mg (Si_2_O_7_) will decrease at the same time, and SFCAM will be formed with CFA, as in the above reaction (7). When the content of MgO increases, the content of MgFe_2_O_4_ decreases gradually with the increase of temperature, with a small amount of decrease, and its ability to form SFCAM by chemical combination decreases. MgO mainly combines Ca_2_Mg (Si_2_O_7_) with CFA and Fe_2_O_3_ to form SFCAM, and the following reaction occurs (8). The increase of MgO content causes high Ca_2_Mg (Si_2_O_7_) content in the mineral phase and inhibits the formation of SFCAM by magnesium ferrite. Therefore, at the temperature range (1000°C–1100°C), MgO is mainly compounded in the form of MgFe_2_O_4_ to form SFCAM. In the high temperature section and low MgO content, MgO is mainly compounded in the form of Ca_2_Mg (Si_2_O_7_) and MgFe_2_O_4_ to form SFCAM; at high temperature section and high MgO content, MgO is mainly compounded in the form of Ca_2_Mg (Si_2_O_7_) to form SFCAM.

(8) $$\begin{array}{c} \text{Fiscalism magnesium silicate}+{\text{Fe}}_{2}{\text{O}}_{3}⟶\text{SFCAM}, \end{array}$$

## 5. RBF Neural Network Model Application

Based on the above experiment of the influence of MgO and Al_2_O_3_ on the formation of composite calcium ferrite, the obtained data are simulated and predicted by an improved RBF neural network model. On the basis of ensuring the prediction accuracy of the model, the formation trend of composite calcium ferrite with different MgO and Al_2_O_3_ additions is further studied, so as to summarize the results of composite calcium ferrite generation with different MgO and Al_2_O_3_ additions in an all-round and multilevel manner. Because the RBF neural network is suitable for the nonlinear changes of the composite calcium ferrite under the addition of different MgO and Al_2_O_3_ and the prediction accuracy is generally high [31], the RBF neural network is selected as the prediction model of the composite calcium ferrite.

### 5.1. RBF Neural Network Model

In the RBF network, the hidden layer performs a fixed nonlinear transformation; *C*_*i*_, *σ*_*i*_, and *ω*_*ik*_ need to be determined through learning and training, which are divided into the three following steps:

(1) The number of hidden layer nodes is determined.
Here we use the resource allocation network (RAN) algorithm to determine the number of hidden layer nodes [32]. As shown in formula (9), the first two input samples initialize the hidden layer nodes of the RBF neural network:
  (9) $$\begin{array}{c} \omega_{0}=y_{1},\omega_{1}=y_{2}-y_{1},c_{1}=x_{2},\sigma_{1}=\mu \delta_{\max}^{2}. \end{array}$$
Judge the change of the node by comparing formulae (10) and (11) with the expected value:
  (10) $$\begin{array}{c} \left|e_{k}\right|=\left|\left|y_{m}\left(k\right)-y\left(k\right)\right|\right|>\varepsilon , \end{array}$$
  (11) di=xi−cnearest=xi−ck1≤k≤Lmin>δi.
Adjust the number of hidden layer nodes according to the distance between the input data and the hidden layer node center. Formula (12) is the parameter value for determining the node:
  (12) $$\begin{array}{c} \omega_{L+1}=e_{k},c_{L+1}=x_{i},\sigma_{L+1}=\gamma d_{i}. \end{array}$$
(2) Determine the center of the basis function *C*_*i*_.
Here, combined with the “K-means clustering method” in fuzzy mathematics to determine the center of the basis function [33], the specific process is as follows:
  (a) Outlier elimination. K-means clustering method is very sensitive to outliers. For this reason, first eliminate data outliers.
  (b) Determine the value of *k*, and the number of clusters *k* is determined by the resource allocation network (RAN) algorithm.
  (c) Take *k* input values as the center of the initial basis function, and perform multiple iterations to update the center of the function according to the principle that objects in the same cluster are close and objects in different clusters are as far away as possible.
(3) Determine width *σ*_*i*_ of the basis function and the connection weight *ω*_*ik*_ from the hidden layer to the output layer.
The basis for selecting the width is to include input data as much as possible, as defined in the following formula:
  (13) $$\begin{array}{c} \sigma_{1}=\sigma_{2}=\ldots =\sigma_{h}=\frac{d_{\max}}{\sqrt{2h}}. \end{array}$$
The connection weight *ω*_*ik*_ is obtained by the pseudoinverse method, as shown in the following equation:
  (14) $$\begin{array}{c} W=G^{+}D. \end{array}$$
The calculation formula of pseudoinverse  *G*^+^ is as follows:
  (15) $$\begin{array}{c} G^{+}={\left(G^{T}G\right)}^{-1}G^{T}. \end{array}$$

Matrix *G* is calculated as follows:

(16) $$\begin{array}{c} gki=\exp\left(-\frac{h}{d_{\max}^{2}}{\left|\left|X_{k}-c_{i}\right|\right|}^{2}\right),\;k=1,2,\ldots ,p;i=1,2,\ldots ,h. \end{array}$$

The weight matrix W is as follows:
  (17) $$\begin{array}{c} \omega =\left\{\omega_{ij}\right\},\;i=1,2,\ldots ,h;j=1,2,\ldots ,n. \end{array}$$

### 5.2. Model Improvement

The pure RBF neural network is easy to fall into the local optimum and make the prediction result error larger. The Dragonfly algorithm (DA) is used to optimize the center of gravity vector, width vector, and weight globally, which can greatly improve the prediction accuracy of the model [34]. The model improvement process is as follows:

1. First determine the number of nodes in the network in order to divide the training set and test set of the data.
2. Initialize the center of gravity vector, width vector, and weight of RBF.
3. Set the step length of the Dragonfly flight, and calculate the parameters of the RBF network by defining the Dragonfly's individual, team, cluster, and foraging and avoiding enemies.
4. Calculate the five behavioral degrees of the Dragonfly.
5. Continuously update the position and step length of the Dragonfly's flight. Carry out loop iteration with the prediction error of the RBF neural network as the fitness function.
6. When the model error meets the requirements, the model iteration ends and the optimal RBF parameters are obtained.

### 5.3. Local Sensitivity Analysis

Local sensitivity analysis is that, for a parameter or for other parameters to take its central value, the amount of change in this parameter each time a change occurs becomes its evaluation model results [35]. There are two methods of variation as follows: the first is the factor variation method (increase or decrease the preanalyzed parameters by 10%); the second is the deviation variation method (increase or decrease the preanalyzed parameters by one standard deviation). A sensitivity coefficient is usually used as a measure of the sensitivity of a parameter. The simplest form of the sensitivity coefficient is

(18) $$\begin{array}{c} S_{i}=\frac{dv}{dp_{i}}, \end{array}$$

where *S*_*i*_ is the sensitivity of the *i*th parameter, *v* is the outcome parameter of the predicted model, and *p*_*i*_ is the *i*th parameter. Of course, some expansions of equation (1) will be made in practical applications.

If the proposed model is insensitive to parameter errors, the conclusion that the model can be applied to different environmental conditions is incorrect. Because a true parameter error can be more than 10% or 20% uncertainty, it can be 2 or 10 times more uncertain, and if the model parameters are not initialized correctly, then the model is insensitive to a 10% change.

### 5.4. Forecast Result Analysis

The experimental data is divided into three mutually exclusive data sets using the set aside method, of which 70% is used as the training set *N*, 20% is used as the test set *T*, and 10% is used as the verification set *V* to predict the generation of calcium ferrite. The improved Dragonfly RBF neural network was used to predict the calcium ferrite generation process, and the prediction accuracy reached 97.6%. The prediction results (Figure 7) are basically consistent with the conclusions obtained from the data analysis and fitting in the previous section, and the accuracy is high, which effectively verifies the correctness of the conclusions of this paper. By comparing the improved Dragonfly RBF neural network prediction with the traditional RBF neural network, it is found that the algorithm being improved has higher prediction accuracy and accelerates the learning of prediction on samples. The local sensitivity analysis shows that the RBF network parameters optimized by the Dragonfly algorithm have little deviation from the model prediction accuracy under 10% change, which is not sensitive. In order to test the robustness of the model, a medical data set published by a certain platform was selected for model prediction. The results showed that the prediction accuracy of the DA-RBF prediction model was also higher than that of the ordinary RBF prediction model, indicating that, for the selection of different data sets, the Dragonfly optimization model can perform a good global optimization of the center of gravity vector, width vector, and weight of the RBF network.

## 6. Energy Spectrum Analysis of Composite Calcium Ferrite Phase Diagram

During the sintering process, MgO reacts with hematite and its gangue components to form a magnesium-rich composite calcium ferrite SFCAM. Studying the reaction process of MgO mineralization to generate SFCAM will help reduce the sinter phase MgO, reduce the content of magnetite, increase the content of calcium ferrite, and improve the performance of the sinter [36].

The energy spectrum analysis was performed on the different mark points of the phase diagram of the composite calcium ferrite ore, and the composition and content were determined. The result data are in Tables 1 and 2. When the temperature is 1200°C, the pore structure is more and the amount of liquid phase is insufficient; meanwhile, at 1250°C, the liquid phase in the mineral phase increases, and the connection between the mineral phases is closer. An acicular calcium ferrite layer is formed around the CA_2_ particles. At this temperature, the reaction of the CFA layer disappears. When the temperature rises by 1250°C, the thickness of the calcium ferrite layer increases, and the small particles of CA_2_ completely react and disappear. A structure with a granular center in the center and a plate-shaped calcium ferrite at the edge are formed, and no magnetite is generated around the CA_2_ particles. In other non-CA_2_ adjacent areas, hematite and silicate form a low-melting liquid phase, producing a large amount of plate-shaped magnetite, but no needle-shaped or plate-shaped calcium ferrite is formed.

Experiments have shown that composite calcium ferrite is generated and grown in the CFA layer [37]. When there is a large amount of composite calcium ferrite around CA_2_ particles, the CFA layer has disappeared. The energy spectrum analysis shows that the composite calcium ferrite produced around CA_2_ has a higher content of magnesium, which is considered to be a magnesium-rich composite calcium ferrite SFCAM. SFCAM is formed between silicate and CA_2_, and the silicate (containing a larger amount of Mg and Fe elements) phases around the outer side of the SFCAM layer and hematite content are lower, indicating that CFA reacts with silicate and hematite to form composite calcium ferrite. In this area, hematite and MgO (in the form of silicate) form composite calcium ferrite. The content of hematite and MgO in the liquid phase is reduced, so no magnetite is formed. In the area without Al_2_O_3_, it is found that silicate reacts with hematite to form a liquid phase, which causes the surrounding hematite to disappear and form a large amount of magnetite. The reaction of silicate and calcium ferrite can generate SFC [38]. The presence of SiO_2_ in calcium ferrite can promote the dissolution of MgO to form compounds. The experimental results show that composite calcium ferrite without aluminum can easily generate magnetite at higher temperatures. XRD detection shows that it can participate in the composite calcium ferrite reaction at a lower temperature. Therefore, no MgFe_2_O_4_ phase is detected at 1200°C and 1250°C.

CFA and CA_2_ are the key reactants for the formation of magnesium-rich composite calcium ferrite SFCAM. The formation of SFCAM mainly takes CA_2_ as the core and is formed by the reaction of CFA with surrounding calcium ferrite and silicate and gradually expands the SFCAM area, increasing the amount of composite calcium ferrite in the mineral phase. MgO participates in the SFCAM formation reaction in the form of silicate and is present in it, which can reduce the content of magnetite. The direct combination of magnesium-containing silicate and hematite will increase the content of magnetite. MgO mainly forms silicate, which is solid-dissolved in magnetite.

## 7. Conclusions and Prospects

1. Al_2_O_3_-2CaO·Fe_2_O_3_ binary system reaction results, the following was found: (1) Al_2_O_3_ reacts with C_2_F at 900°C–950°C to form CA_2_ and CF, and CFA is formed at the CA_2_/CF interface. (2) As the temperature increases, the ability of Al^3+^ to pass through the CA_2_ layer is less than that of Ca^2+^ to pass through the CF and CFA layers. Ca^2+^ diffuses through the CF and CFA forming layers to the CA/CA_2_ interface, and CA_2_ decomposes to form CA. (3) The temperature of CA generation is high, and it cannot participate in the generation of CFA. The chemical formula of the average content of each element in CFA is Ca_1.5_Fe_1.6_Al_1.6_O_5.0_, which is close to 2CaO·Fe_2_O_3_·Al_2_O_3_.
2. In the sintering process of the C_2_F-Al_2_O_3_-Fe_2_O_3_ ternary system: (1) Ca^2+^ ions at the C_2_F/CFA interface diffuse to the CA_2_/CFA interface and are dissolved by CFA but do not diffuse to the CA_2_ interface. Fe_2_O_3_ can improve the solubility of CFA to CaO. (2) Fe_2_O_3_ can form CFA and CA_2_ with Al_2_O_3_ and C_2_F at around 950°C. The reaction mechanism is that first Al_2_O_3_ reacts with C_2_F to form CA_2_ and CF, and then CA_2_, CF, and Fe_2_O_3_ react to form CFA.
3. During the sintering experiment of the CaO (CaCO_3_)-Al_2_O_3_-Fe_2_O_3_ ternary system: (1) the reaction first generates dicalcium ferrite 2CaO·Fe_2_O_3_ and hemicalcium aluminate CA_2_, forming a CA_2_/C2F interface. (2) C_2_F reacts with Fe_2_O_3_ at around 800°C to produce ferrite monocalcium CaO·Fe_2_O_3_, and the C_2_F/CA_2_ interface transforms into the CF/CA_2_ interface. CF and CA_2_ at the interface between 850°C and 900°C react with Fe_2_O_3_ in the mineral phase to generate CFA.
4. Al_2_O_3_ mainly promotes the conversion of calcium ferrite to composite calcium ferrite. A coating layer of CA_2_ and CFA products is formed around Al_2_O_3_. CFA is formed around the CA_2_ layer. The CFA formation reaction in the ternary CaO(CaCO_3_)-Al_2_O_3_-Fe_2_O_3_ system is the easiest to proceed.
5. MgO behavior in the formation mechanism of magnesium-rich composite calcium ferrite: When the content of MgO is low, MgO promotes the formation of magnesium-rich composite calcium ferrite in the form of calcium magnesium silicate and ferrite; when the content of MgO is high, MgO mainly promotes the formation of magnesium-rich composite calcium ferrite in the form of calcium-magnesium silicate. At high temperature and high MgO content, MgO promotes the decomposition of magnesium-rich composite calcium ferrite to generate magnetite.
6. The composite calcium ferrite is formed at the edge of the CFA layer and is formed by the reaction of CFA, magnesium ferrite, calcium magnesium silicate, and hematite until the nuclear reaction of CFA and CA_2_ shrinks and disappears completely to form a composite calcium ferrite generating area. The composite calcium ferrite generated near the CFA area is not easy to decompose to form magnetite. CFA can inhibit the escape of MgO in the composite calcium ferrite; the MgO in the magnesium-rich composite calcium ferrite far away from the CFA area is easy to escape, which promotes the decomposition of the magnesium-rich composite calcium ferrite to generate magnetite.
7. Data preprocessing, data correlation analysis, and data fitting analysis are performed on the obtained data through intelligent algorithms, and, combined with the energy spectrum analysis of the composite calcium ferrite phase diagram, the influence of MgO and Al_2_O_3_ on the formation of composite calcium ferrite is obtained. In the next work, the intelligent prediction algorithm will be used to study the formation trend of composite calcium ferrite and further analyze the influence of MgO and Al_2_O_3_ on the formation of composite calcium ferrite.
8. Establish a DA-RBF neural network model, and use the Dragonfly algorithm to improve the model. Use the model to predict the calcium ferrite generation process. Compared with the traditional RBF neural network model, the DA-RBF network model can better optimize the center of gravity vector, width vector, and weight of the RBF network globally, reducing the prediction error, and it has a good generalization ability.
9. The DA-RBF model has good predictive performance and generalization ability. However, the model cannot explain its own reasoning process well. Therefore, in the following model study, the physicochemical mechanism during the sintering process will be further explored based on the DA-RBF model of MgO and Al_2_O_3_ composite calcium ferrite formation mechanism.

## Figures and Tables

**Figure 1:** Interface reaction schematic.

**Figure 2:** Al_2_O_3_-CaO-Fe_2_O_3_ XRD diagrams of phase.

**Figure 3:** Effect of Al_2_O_3_ content on phase XRD. (a) Fe_2_O_3_(PDF: 16-0653); (b) SFCA-I(PDF: 52-1258); (c) C_4_F_7_(PDF: 13-0395); (d) C_2_F(PDF: 89-8669); (e) CA_2_(PDF: 89-3851); (f) CaAl_2_Fe_4_O_10_(PDF: 21-0830).

**Figure 4:** XRD diagrams of phase (w(MgO) = 1.3%).

**Figure 5:** Diffraction peak integral intensity; temperature curve of phase with different MgO content. (a) w(MgO) = 1.3%; (b) w(MgO) = 2.6%; (c) w(MgO) = 3.9%; (d) SFCAM integral intensity.

**Figure 6:** Comparison chart of fitting algorithm.

**Figure 7:** Improved RBF neural network algorithm for Dragonfly prediction.

**Table 1:** Determination of elemental content of phase F37-2 (atom%).

	O-K	Mg-K	Al-K	Si-K	Ca-K	Fe-K
pt1	55.86		1.27	3.72	2.92	36.23
pt2	51.09	4.42	5.95	14.03	12.54	11.97
pt3	53.69	1.84	26.87	3.40	6.95	7.24
pt4	45.74	3.96	9.09	7.92	7.66	25.90
pt5	55.24	0.30	34.31		9.44	0.71

**Table 2:** Determination of elemental content of phase F38-2 (atom%).

	O-K	Mg-K	Al-K	Si-K	Ca-K	Fe-K
pt1	50.05		1.58			48.36
pt2	59.90		1.64		0.39	38.07
pt3	51.41	1.44	4.16	17.51	17.68	7.81
pt4	48.50	4.81	7.80	6.94	8.26	23.69

## Data Availability

The data and images used to support the findings of this study were obtained through enterprises and laboratories, and no external data were used for research. As part of the data comes from enterprises, the data cannot be disclosed.
